The article "Proton Pump Inhibitor Use and Magnesium Concentrations in Hemodialysis Patients: A Cross-Sectional Study" was published in 2015. Journal: PLoS One.

# Proton Pump Inhibitor Use and Magnesium Concentrations in Hemodialysis Patients: A Cross-Sectional Study

**DOI:** 10.1371/journal.pone.0143656

**Published:** 2015-11-30

**Authors:** Akio Nakashima, Ichiro Ohkido, Keitaro Yokoyama, Aki Mafune, Mitsuyoshi Urashima, Takashi Yokoo

**Affiliations:** 1 Division of Nephrology and Hypertension, Department of Internal Medicine, Jikei University School of Medicine, Tokyo, Japan; 2 Division of Molecular Epidemiology, Jikei University School of Medicine, Tokyo, Japan; Hospital Universitario de La Princesa, SPAIN

## Abstract

Magnesium concentration is a proven predictor of mortality in hemodialysis patients. Recent reports have indicated that proton pump inhibitor (PPI) use affects serum magnesium levels, however few studies have investigated the relationship between PPI use and magnesium levels in hemodialysis patients. This study aimed to clarify the association between PPI use and serum magnesium levels in hemodialysis patients. We designed this cross sectional study and included 1189 hemodialysis patients in stable condition. Associations between PPI and magnesium-related factors, as well as other possible confounders, were evaluated using a multiple regression model. We defined hypomagnesemia as a value < 2.0 mg/dL, and created comparable logistic regression models to assess the association between PPI use and hypomagnesemia. PPI use is associated with a significantly lower mean serum magnesium level than histamine 2 (H2) receptor antagonists or no acid-suppressive medications (mean [SD] PPI: 2.52 [0.45] mg/dL; H2 receptor antagonist: 2.68 [0.41] mg/dL; no acid suppressive medications: 2.68 [0.46] mg/dL; *P* = 0.001). Hypomagnesemia remained significantly associated with PPI (adjusted OR, OR: 2.05; 95% CI: 1.14–3.69; *P* = 0.017). PPI use is associated with an increased risk of hypomagnesemia in hemodialysis patients. Future prospective studies are needed to explore magnesium replacement in PPI users on hemodialysis.

## Introduction

Magnesium is known to play an important role in biological processes, including regulation of enzymatic activity, protein synthesis, membrane stabilization, and regulation of ion channels [1]. Recently, magnesium abnormalities have been reported as one of the predictors of mortality in hemodialysis (HD) patients [2]. Hypomagnesemia has been implicated in hypertension [3], type 2 diabetes mellitus [4], atrial fibrillation [5], and sudden cardiac death [6]. In addition, disordered bone metabolism is also associated with magnesium abnormalities [7].

Proton pump inhibitors (PPIs) are widely prescribed throughout the world, including for HD patients. PPIs are easy to prescribe for HD patients because PPIs undergo extensive hepatic metabolism, so there is no need to adjust the dosage of various concomitant medications that the patient might be receiving, such as histamine-2 (H2) receptor antagonists. Recent reports have shown that the use of PPI induces hypomagnesemia [8]. Nevertheless, fewer than 30 cases of severe hypomagnesemia in patients on PPI therapy have been reported since 2006 [9]. On March 2, 2011, the U.S. Food and Drug Administration (FDA) issued a drug safety alert that long-time PPI use may cause low levels of serum magnesium.

The article "Proton Pump Inhibitor Use and Magnesium Concentrations in Hemodialysis Patients: A Cross-Sectional Study" was published in 2015. Journal: PLoS One.

Previous case reports and studies that examined the association of PPI use with serum magnesium levels in patients with normal kidney function have excluded patients with end-stage renal disease (ESRD). Therefore, the aim of the present study was to examine the relationship between PPI use and serum magnesium concentrations in HD patients. Former observational studies have suggested that an association of PPI use with hypomagnesemia was found in patients taking diuretics rather than in the general population or ICU patients [10]. Thus, another aim of the present study was to evaluate the effect of diuretics on low magnesium concentrations in connection with PPI use in dialysis patients.

## Methods

### Study population

We recruited HD patients from 15 dialysis units between May 2012 and June 2013. The patients were over 20 years old, and at least 3 months had elapsed since they started dialysis therapy. All patients received dialysis 3 times weekly (3–5 h/session). We excluded patients with acute bleeding, acute cardiovascular disease, liver dysfunction, and infection at baseline. Patients who were prescribed magnesium were also excluded. Ultimately, we analyzed 1189 patients. The study protocol was reviewed and approved by the Jikei Institutional Review Board at Jikei University School of Medicine (22–182 6359). All study procedures were in accordance with the Declaration of Helsinki and its revisions. Signed informed consent was obtained from all patients prior to inclusion in the study.

In all dialysis centers that participated in this study, the magnesium composition of the dialysate utilized was 1.0 mEq/L.

### Laboratory analysis and clinical information

Blood pressure and heart rate were measured before each dialysis session. Blood samples were collected before the HD session after the longest interdialytic period. Routine biochemical measurements included magnesium, potassium, phosphorus, calcium, serum albumin, blood urea nitrogen, alkaline phosphatase, creatinine, hemoglobin, intact parathyroid hormone (PTH), and C-reactive protein (CRP). The dose of delivered dialysis was measured by single pool Kt/V.

The article "Proton Pump Inhibitor Use and Magnesium Concentrations in Hemodialysis Patients: A Cross-Sectional Study" was published in 2015. Journal: PLoS One.

Age, sex, dialysis vintage, primary illness of kidney dysfunction, and past medical history were extracted from medical records. Medication information (use of PPI, H2 receptor antagonist, diuretic, antiplatelet drug, vitamin K antagonist, phosphate binder, vitamin D receptor antagonist, cinacalcet, antihypertensive medication, and so on) was taken from prescription records.

### Statistical analysis

Non-normally distributed data were expressed as median (range), and normally distributed data were summarized as mean ± SD as appropriate. Binary data were summarized as percentages. Statistical significance was set at *P*<0.05.

We categorized patients by baseline characteristics according to use of PPI, H2 receptor antagonists, or no acid suppressive medication. The chi-square test or two-sample *t*-test was used to assess patients’ characteristics as appropriate.

Associations between PPI and magnesium-related factors, as well as other possible confounders, were evaluated using a multiple regression model. Age, blood pressure, and laboratory values were all included as continuous variables. Model I included age, sex, and dialysis vintage. Model II included the factors in Model I with the addition of systolic blood pressure, body mass index (BMI), comorbidities (diabetes mellitus, atrial fibrillation, gastric hemorrhage, cerebral infarction, and ischemic heart disease), medications (diuretic, antiplatelet drug, vitamin K antagonist, phosphate binder, vitamin D receptor antagonist, cinacalcet, and antihypertensive medication), serum albumin, serum potassium, serum calcium, serum phosphate, iPTH, Kt/V, and CRP.

To elucidate the dose-dependent effect of PPI exposure on hypomagnesemia, we also defined high-dose PPI use and low-dose PPI use as follows: high-dose use included lansoprazole 30 mg, omeprazole 20 mg, rabeprazole 20 mg, and esomeprazole 20 mg; low-dose use included lansoprazole 15 mg, omeprazole 10 mg, rabeprazole 10 mg, and esomeprazole 10 mg.

To compare the effects on magnesium levels between use of PPIs and use of H2 receptor antagonists, we created binary indicator variables for PPI or H2 receptor antagonist use. Differences between the two groups’ magnesium concentrations were assessed by the analysis of variance (ANOVA) test.

We defined hypomagnesemia as a value < 2.0 mg/dL, and created comparable logistic regression models to assess the association between PPI use and hypomagnesemia. Because HD patients have a tendency to become hypermagnesemic, whereas hypomagnesemia, defined as a serum level < 1.8 mg/dL is relatively uncommon (< 1%), and typically observed in association with hypokalemia and hypophosphatemia, we adopted hypomagnesemia as a value < 2.0 mg/dL. The same variables used in the multivariate linear regression analysis (Model II) were included without further dichotomization.

The article "Proton Pump Inhibitor Use and Magnesium Concentrations in Hemodialysis Patients: A Cross-Sectional Study" was published in 2015. Journal: PLoS One.

Finally, the effects of diuretic use and dialysis vintage on magnesium levels in HD patients who received PPIs were analyzed by regression models. We used the same variables used in the multivariate linear regression (Model II). As HD patients who have undergone dialysis therapy > 24 months are usually anuric, we analyzed patients who had a shorter dialysis vintage (< 24 months) as an alternative for evaluating residual renal function.

All statistical analyses were performed using STATA 13.0 (STATA Corp., College Station, TX, USA).

## Results

### Patient characteristics

The study population consisted of 1189 patients with a mean age of 63.5 ± 11.8 years; 70.1% were men, and the mean dialysis vintage was 109.9 ± 92.1 months. As shown in Table 1, 52.3% of the study patients were PPI users, and 12.1% were H2 receptor antagonist users. There were no patients who were prescribed both a PPI and an H2 receptor antagonist. The PPI users had a mild tendency to be older, received higher doses of antiplatelet drugs, and had a higher rate of comorbidities. Diuretic use was uncommon among both PPI users and the H2 receptor antagonist users; there was no significant difference in the diuretic ratio. The mean serum magnesium level of the subjects was 2.6 ± 0.5 mg/dL.

**Table 1:** Patient characteristics.

	Proton pump inhibitor (n = 623)	H2 receptor antagonist (n = 128)	No acid suppressive medications (n = 438)	*P* value
Age mean (s.d.), years	64.5±10.8	63.5±11.7	62.0±12.6	0.003
Male sex, (%)	426 (68.4)	89 (70.1)	318 (72.6)	0.335
Dialysis vintage mean (s.d.), years	112.6±96.5	100.4±65.6	108.8±92.3	0.382
Body mass index mean (s.d.)	22.2	22.0	22.2	0.89
Systolic blood pressure mean (s.d.), mmHg	151±22	157±22	152±23	0.025
Diastolic blood pressure mean (s.d), mmHg	79±14	84±14	79±14	0.002
*Past medical history (%)*				
Diabetes mellitus	255 (41.1)	44 (34.7)	148 (34.0)	0.05
Ischemic heart disease	159 (25.5)	19 (14.8)	35 (8.0)	<0.001
Cerebral infarction	85 (13.6)	19 (14.8)	37 (8.5)	0.02
Gastric hemorrhage	124 (19.9)	17 (13.3)	36 (8.2)	<0.001
Atrial fibrillation	76 (12.2)	15 (11.7)	46 (10.5)	0.694
Medications (%)				
Aspirin	307 (49.3)	52 (40.6)	130 (29.7)	<0.001
Cilostazol	51 (8.2)	7 (5.8)	28 (6.4)	0.387
Clopidogrel	74 (11.9)	12 (9.4)	19 (4.3)	<0.001
Vitamin K antagonist	61 (9.8)	11 (8.6)	25 (5.7)	0.056
Vitamin D receptor antagonist	417 (66.9)	62 (48.4)	280 (63.9)	<0.001
ACE-I or ARB	332 (54.5)	52 (40.9)	217 (51.4)	0.02
Furosemide	148 (23.8)	29 (22.7)	114 (26.0)	0.614
Laboratory measurements				
Hemoglobin (g/dL)	10.4±1.0	10.6±1.0	10.6±1.1	0.037
Albumin (g/dL)	3.7±0.3	3.7±0.4	3.8±0.3	0.054
Blood urea nitrogen (mg/dL)	63.4±14.4	66.03±14.79	67.46±13.75	<0.001
Creatinine (mg/dL)	11.24±2.87	12.38±3.43	11.98±3.29	<0.001
Sodium (mEq/L)	139.0±3.0	138.7±3.0	139.2±2.7	0.298
Potassium (mEq/L)	4.98±0.73	4.99±0.73	5.03±0.68	0.559
C-reactive protein (mg/dL)	0.57±1.39	0.49±1.10	0.41±1.70	0.264
Kt/V	1.40±0.27	1.40±0.25	1.38±0.24	0.435
Alkaline phosphatase (IU/L)	252±126	222±89	232±118	0.009
Calcium (mg/dL)	8.8±0.6	9.0±0.6	9.0±0.7	<0.001
Phosphorus (mg/dL)	5.5±1.4	5.7±0.6	5.5±1.3	0.293
Parathyroid hormone (pg/mL)	173±127	111±181	181±166	0.009

*P* values reflect group across differences. Abbreviations: H2,histamine 2; ACE-I, angiotensin converting enzyme inhibitor; ARB, angiotensin II receptor blocker. Conversion factors for units: serum creatinine in mg/dL to mol/L, *88.4; blood urea nitrogen in mg/dL to mmol/L,*0.357; Calcium in mg/dL to mmol/L,*0.2495; Phosphorus in mg/dL to mmol/L, *0.3229.

The article "Proton Pump Inhibitor Use and Magnesium Concentrations in Hemodialysis Patients: A Cross-Sectional Study" was published in 2015. Journal: PLoS One.

### Relationship of PPI use to magnesium concentration

As shown in Table 2, among the study patients, PPI users had significantly lower mean serum magnesium levels in unadjusted analysis than H2 receptor antagonists users and patients receiving no acid medication (mean [SD] PPI: 2.52 [0.45] mg/dL; H2 receptor antagonist: 2.68 [0.41] mg/dL; no acid suppressive medications: 2.68 [0.46] mg/dL; *P* = 0.001). In addition, after adjusting for patient background (Model I), and in the fully adjusted model (Model II), PPI exposure was significantly related to lower magnesium concentration in comparison with H2 receptor antagonist users and patients receiving no acid medication.

**Table 2:** Associations between serum magnesium levels and Proton Pump inhibitor use as determined by regression analyses.

	Proton Pump inhibitor						H2 receptor antagonist		No acid-suppressive medications
	Total		Low-dose proton pump inhibitors		High-dose proton pump inhibitors				
Magnesium±s.e. (mg/dL)	2.52±0.46		2.54±0.47		2.47±0.39		2.68±0.4		2.68±0.45
	β-coefficient±s.e.	*P* value	β-coefficient±s.e.	*P* value	β-coefficient±s.e	*P* value	β-coefficient±s.e	*P* value	Reference
Unadjusted model	-0.155±0.026	<0.001	-0.141±0.028	<0.001	-0.210±0.043	<0.001	-0.129±0.0451	0.775	-
Model I	-0.146±0.026	<0.001	-0.135±0.0283	<0.001	-0.204±0.042	<0.001	-0.143±0.0446	0.748	-
Model II	-0.147±0.029	<0.001	-0.131±0.031	<0.001	-0.185±0.046	<0.001	-0.181±0.0472	0.711	

Reference category is the patients on no acid suppressive medications. β-coefficients ± s.e’s and *P* values are provide for each variable. Model I includes age, dialysis vintage and sex. Model II includes all variables in Model I and the addition of Diabetes mellitus, Kt/V, systolic blood pressure, albumin, potassium, C-reactive protein, sodium, blood urea nitrogen, parathyroid hormone, phosphorus, calcium, hemoglobin, furosemide, antiplatelet drug, vitamin K antagonist, angiotensin converting enzyme inhibitor or angiotensin II receptor blocker, phosphate binder, vitamin D receptor antagonist, atrial fibrillation, gastric hemorrhage, cerebral infarction, and ischemic heart disease. Conversion factors for units: serum magnesium in mg/dL to mol/L, *0.4114.

The article "Proton Pump Inhibitor Use and Magnesium Concentrations in Hemodialysis Patients: A Cross-Sectional Study" was published in 2015. Journal: PLoS One.

We also analyzed high-dose PPI use, low-dose PPI use, and no PPI use with respect to serum magnesium levels. In the unadjusted model, there were significant dose-dependent effects of PPI on serum magnesium levels (mean [SD] high-dose PPI: 2.47 [0.39] mg/dL; low-dose PPI: 2.53 [0.47] mg/dL; no PPI: 2.68[0.44] mg/dL; *P* < 0.001). Using multiple linear regression analysis with magnesium concentration as the dependent variable, the effect of PPI dose was significantly associated with lower magnesium concentration in the adjusted models (Model I, Model II).

### Relationship of PPI use to hypomagnesemia

Hypomagnesemia, defined as a serum magnesium level < 2.0 mg/dL, was found in 104 of the 1189 HD patients. PPI use was associated with a higher prevalence of hypomagnesemia (PPI: 11.2% [70/623]; H2 receptor antagonist: 7.0% [9/128]; no acid suppressive medications: 5.7% [25/438]). As shown in Table 3, logistic regression analysis was performed for PPI use and hypomagnesemia after adjustment for the same values used in the multivariate linear regression analysis (Model II). PPI exposure remained significantly associated with hypomagnesemia (either by the unadjusted or adjusted model, adjusted OR, 2.05; 95% CI, 1.14–3.69 *P* = 0.017). Both low-dose and high-dose PPI use were significantly associated with hypomagnesemia in a dose-dependent manner. Multiple logistic regression analysis also revealed that age, BMI, and serum albumin, were risk factors for hypomagnesemia in HD patients.

**Table 3:** Logistic analysis between Proton Pump inhibitor use and hypomagnesemia.

		Odds ratio	95% CI	*P* value
Unadjusted	Proton pump inhibitor	1.98	1.30–3.03	<0.001
	Low-dose	1.80	1.15–2.84	<0.001
	High-dose	2.67	1.47–4.87	<0.001
Adjusted	Proton pump inhibitor	2.05	1.14–3.69	0.017
	Low-dose	2.01	1.11–3.89	0.02
	High-dose	2.99	1.10–8.42	0.02
	Body mass index	1.16	1.02–1.41	0.04
	Albumin	0.24	0.09–0.6	0.003
	Age	0.97	0.91–1.01	0.097
	Sex	1.41	0.52–6.7	0.53
	Diabetes mellitus	0.28	0.18–1.79	0.36

Hypomagnesemia is defined as ≤ 2.0 mg/dL (0.82mmol/L). Adjusted models includes age, dialysis vintage, sex, Diabetes mellitus, Kt/V, systolic blood pressure, albumin, potassium, C-reactive protein, sodium, blood urea nitrogen, parathyroid hormone, phosphorus, calcium, hemoglobin, furosemide, antiplatelet drug, vitamin K antagonist, angiotensin converting enzyme inhibitor or angiotensin II receptor blocker, phosphate binder, vitamin D receptor antagonist, atrial fibrillation, gastric hemorrhage, cerebral infarction, and ischemic heart disease.

The article "Proton Pump Inhibitor Use and Magnesium Concentrations in Hemodialysis Patients: A Cross-Sectional Study" was published in 2015. Journal: PLoS One.

### Relationship between PPI use and diuretic use or dialysis vintage and magnesium levels

We analyzed whether diuretic use and shorter dialysis vintage (< 24 months) affected magnesium concentrations with PPI use. As seen in Table 4, the effect of PPI exposure on magnesium levels was not individually altered by the use of diuretics or shorter dialysis vintage. The combination of diuretic use and dialysis vintage < 24 months also did not affect the magnesium concentration among the patients who took PPIs.

**Table 4:** Effect of diuretic use and hemodialysis vintage on association between acid suppressive therapy and serum magnesium.

	Proton pump inhibitor		H2 receptor antagonist		No acid-suppressive medications
	β-coefficient±s.e.	*P* value	β-coefficient±s.e.	*P* value	reference
Furosemide (n = 291)	-0.054±0.047	0.249	0.006±0.085	0.565	-
Shorter dialysis vintage <24 mo (n = 188)	0.069±0.082	0.421	0.017±0.126	0.984	-
Furosemide+shorter dialysis vintage <24 mo(n = 96)	0.0139±0.092	0.778	0.142±0.19	0.41	-

Abbreviation: H2, histamine-2. Reference category is patients on no acid-suppressive medications. β-coefficients ± s.e’s and *P* values are provided for each variable. Adjusted models includes age, dialysis vintage, sex, Diabetes mellitus, Kt/V, systolic blood pressure, albumin, potassium, C-reactive protein, sodium, blood urea nitrogen, parathyroid hormone, phosphorus, calcium, hemoglobin, furosemide, antiplatelet drug, vitamin K antagonist, angiotensin converting enzyme inhibitor or angiotensin II receptor blocker, phosphate binder, vitamin D receptor antagonist, atrial fibrillation, gastric hemorrhage, cerebral infarction, and ischemic heart disease.

## Discussion

The present study results showed that PPI exposure is associated with magnesium levels and hypomagnesemia in HD patients, and that this effect of PPI is dose-dependent. The strength of the relationship between hypomagnesemia and PPI remained robust and independent of underlying comorbidities. Diuretic use and shorter dialysis vintage < 24 months were not associated with hypomagnesemia due to PPI use in HD patients. Although former studies have suggested a relationship between PPI use and hypomagnesemia in ICU patients [10] or the general population [11], the present study is the first to have a sufficiently large study population among stable HD patients to analyze the effect of PPI use on magnesium concentration and suggest that PPI exposure is associated with hypomagnesemia in HD patients.

The article "Proton Pump Inhibitor Use and Magnesium Concentrations in Hemodialysis Patients: A Cross-Sectional Study" was published in 2015. Journal: PLoS One.

The most common causes of acquired hypomagnesemia in HD patients are general malnutrition, diarrhea, malabsorption syndrome, primary aldosteronism, and alcohol consumption [12]. An inadequate dialysate magnesium concentration can also induce hypomagnesemia [13]. However, it is difficult to improve the magnesium concentration in HD patients. The serum magnesium concentration depends mainly on the balance between gastrointestinal absorption and renal excretion [14] by both active transcellular and passive paracellular mechanisms. Regarding gastrointestinal absorption, passive reabsorption is paracellularly regulated by the enterocyte tight junction proteins claudin-16 and claudin-19, [15], which are responsible for approximately 90% of the absorption [16]. Passive intestinal absorption is dependent on low affinity and concentration. On the other hand, an active transcellular process is mediated by transport channels, and by transient receptor potential melastatins -6 and -7 (TRPM6/7), which are present in the apical membranes of the enterocytes [17]. Magnesium excretion is regulated tightly by TRPM6 in the renal distal convoluted tubules.

The mechanism of hypomagnesemia caused by PPI exposure has gradually come to be understood. Almost all case series studies of hypomagnesemia resulting from PPI treatment have reported that urine magnesium levels were low [18]. Additionally, a recent study suggested that PPI use is associated with lower urinary magnesium excretion [19]. Former studies have indicated that PPI does not induce urinary magnesium loss. It has recently been advocated that intestinal malabsorption of magnesium is the main cause of PPI-related hypomagnesemia. Because PPIs inhibit H+/K+-ATPase activity in the gastrointestinal tract, this inhibition reduces the intestine luminal pH to 0.5 and changes the TRPM6/7 channel affinity for Mg^2^+ [20]. In an *in vivo* mouse model, omeprazole feeding did not change the serum magnesium level or the amount of urinary magnesium excretion. However, the mRNA expression level of TRPM6 and H+/K+-ATPase in the colon increased, and little or no change occurred in the kidney [21]. The authors hypothesize that as omeprazole inhibits H+/K+-ATPase activity, resulting in reduced excretion of protons into the intestine, this effect impairs TRPM6-mediated Mg^2^+absorption stimulated by extracellular protons [21]. As a result, the mRNA expression level of TRPM6 in the intestine increases in parallel.

In HD patients, the prevalence of gastrointestinal disease is higher than in the general population. Patients with ESRD often have gastrointestinal complications, for example, gastroesophageal reflux, gastritis, gastrointestinal bleeding ulcers, and nausea [22]. The prevalence of gastrointestinal symptoms in dialysis patients is thought to range from 70–90% [23]. The percentage of dialysis patients who receive PPIs is increasing because of such gastrointestinal conditions. In addition, HD patients usually have several comorbidities, such as ischemic heart disease, cerebral infarction, and peripheral arterial disease, and these diseases result in a high prevalence of ESRD patients taking antiplatelet drugs [24]. As a result, PPIs are administered to ESRD patients prophylactically to prevent gastrointestinal bleeding [25]. According to data from the Dialysis Outcomes and Practice Patterns Study (DOPPS), the proportion of patients prescribed either a PPI or an H2 receptor antagonist was 36–38%, with a concomitant increase in the use of PPIs [26]. Physicians need to pay more attention to PPI use in dialysis patients than previously. One study in HD patients found that long-term PPI use is associated with vascular calcification [27].

The article "Proton Pump Inhibitor Use and Magnesium Concentrations in Hemodialysis Patients: A Cross-Sectional Study" was published in 2015. Journal: PLoS One.

There are several risk factors for vascular calcification: hyperphosphatemia, hypercalcemia, hyperparathyroidism, vitamin D abnormality, and warfarin use [28]. As the dialysis patients who are prescribed a PPI may have several comorbidities and eat a small amount because of gastrointestinal disorders, they tend to be vitamin D deficient. Low levels of vitamin D increase TNF-α levels and decrease IL-10 levels [29] because TNF-α worsens intimal atherosclerosis and vascular calcification and IL-10 has antiatherogenic properties [30]. Because of the high incidence of atrial fibrillation and valvular disease, patients with dialysis are more likely to be taking warfarin [31]. Warfarin blocks vitamin K-dependent proteins such as matrix Gla protein (MGP) and growth arrest-specific gene 6 (Gas-6), which are important inhibitors of mineralization [32]. Warfarin promotes aortic stenosis and excessive vascular calcification [33].

In addition, dialysis patients who are prescribed PPIs have a high prevalence of vascular calcification, especially with warfarin use [27]. A recent study also reported that hypomagnesemia causes vascular calcification in human aortic vascular smooth muscle cells [34]. We should pay attention to vascular calcification in HD patients who use PPIs and warfarin.

Another study reported that PPI users have lower bone mineral density values [35].A previous study also showed that PPI use is a risk factor of hip fracture in the general population [36]. The advocated mechanism is that PPIs inhibit calcium absorption in the intestine and directly suppress bone formation [37]. In addition, hypomagnesemia is also a risk factor for fracture [7]. Magnesium deficiency causes an increased rate of hydroxyapatite formation, resulting in larger crystals and lower bone mass and brittle bones [38]. In addition, magnesium has an effect on osteoblast activity and osteoclast number through a nitric oxide-dependent mechanism and affects bone metabolism through altered calcium homeostasis via influences on calcium transport and urinary retention [39].

The article "Proton Pump Inhibitor Use and Magnesium Concentrations in Hemodialysis Patients: A Cross-Sectional Study" was published in 2015. Journal: PLoS One.

A prior study reported that among a sample of critically ill patients, the combination of PPI use and diuretic exposure was associated with hypomagnesemia [10]. Because PPIs prevent magnesium absorption in the gastrointestinal tract, the upregulation of renal tubular magnesium reabsorption works in a complementary manner to maintain magnesium balance. Because diuretic agents usually cause magnesium excretion through the renal tubules, it is possible that diuretic use accelerates hypomagnesemia in patients receiving PPI therapy. The present study results do not support the exacerbation of hypomagnesemia by the combination of PPI and diuretics. One reason is that our study population consisted of HD patients with a mean dialysis vintage of 109.9 months. In general, dialysis patients develop oliguria if their dialysis vintage is longer than 2 years [40]. In addition to a reduction in urine volume, the urinary solute of these patients also decreases despite the use of diuretics [41]. Even though HD patients use PPIs, no effects of furosemide on magnesium concentrations have been observed because of the decline in residual renal function. A previous study that investigated the relationship between PPI use and hypomagnesemia among HD patients reported that administration of furosemide is a risk factor for hypomagnesemia [42]. However, because the study population of the former study was different from that of our study with respect to dialysis vintage (41.2 vs 109.9 months), the discrepancy could be attributed to residual renal function. The present study did not examine urinary volume or analyze urinary electrolytes. A further well-designed study on these topics is needed.

Although most of the former studies that investigated the magnesium levels and PPI use in the general population defined hypomagnesemia as < 1.8mg/dL, we defined hypomagnesemia as < 2.0mg/dL. Sakaguchi et al reported higher all-cause and cardiovascular mortality in HD patients in the lowest magnesium sextile (< 2.3 mg/dL) [2]. Even though magnesium absorption from the intestine is found to be impaired in patients with kidney failure, HD patients have a tendency to become hypermagnesemic. Because of anuria and dialysate concentration, serum magnesium level < 1.8 mg/dL is relatively uncommon (<1%) and is typically observed in association with hypokalemia and hypophosphatemia [43]. Due to the above reasons, we set hypomagnesium as < 2.0 mg/dL in our study of HD patients.

The article "Proton Pump Inhibitor Use and Magnesium Concentrations in Hemodialysis Patients: A Cross-Sectional Study" was published in 2015. Journal: PLoS One.

Although our study showed that PPI use is a risk factor of hypomagnesemia in HD patients, age, albumin, and body mass index were also significantly associated with hypomagnesemia. Age, albumin, and body mass index might reflect malnutrition, frailty, insufficient diet, and other comorbidities. On the other hand, our results did not show an association of hypomagnesemia with potassium, phosphate, and parathyroid hormone concentration. The mechanisms that have been proposed suggest that potassium affects the renal tubules and promotes magnesium excretion in the kidney [44,45]. Hyperphosphatemia and hyperparathyroidism also promote magnesium excretion [46]. However, the influence of potassium, phosphate, and parathyroid hormone on magnesium concentration was not seen in this study. In our study, because there were the few patients with a shorter dialysis vintage (< 24 months, n = 188) who might have had residual kidney function, electrolyte and parathyroid hormone levels might not have affected magnesium concentration.

The present study had several limitations. First, because this was a cross-sectional study, the association found between PPI exposure and hypomagnesemia could not establish causality. Second, information was not available on the length of PPI exposure. Past reports have shown that long-term PPI treatment is a risk factor for hypomagnesemia [9]. However, another study reported that short-term PPI use (14 days) also induced hypomagnesemia [47]. The third limitation of the present study is that data on residual kidney function and urinary Mg excretion were not available. Several studies have shown that combination treatment using a PPI and diuretic agents induces hypomagnesemia in ICU patients. However, the results of the present study showed no relationship between PPI use and furosemide. The fourth limitation of the present study was that information on daily magnesium intake was not obtained. Former studies have reported that dietary magnesium repletion can correct serum concentrations [48] but not in all cases [49].The fifth limitation is that our study did not have information about dietary intake. It is possible that patients who were prescribed a PPI had more gastrointestinal symptoms and had a lower dietary intake than those taking an H2-blocker. Because in this study there was a significant difference in magnesium concentrations between PPI users and H2-blocker users, magnesium intake is the unknown confounder.

The article "Proton Pump Inhibitor Use and Magnesium Concentrations in Hemodialysis Patients: A Cross-Sectional Study" was published in 2015. Journal: PLoS One.

Further interventional studies are needed to elucidate whether there is a cause-and-effect relationship between hypomagnesemia and PPI use; and such studies should evaluate urine volume and urine magnesium concentration. At present, we propose that in dialysis patients who are prescribed a PPI, physicians should monitor serum magnesium levels and switch from the PPI to an H2 receptor antagonist or adjust the dose of the PPI if hypomagnesemia is confirmed.

In conclusion, PPI use has been associated with the mean serum magnesium levels and hypomagnesemia in HD patients. However, the present study results imply that the combination of PPI and diuretic use in HD patients is not associated with magnesium level or risk for hypomagnesemia. A future prospective study is required to clarify the need for magnesium replacement among HD patients who are PPI users, and elucidate the underlying mechanisms.
